This article has been retracted.

# Microorganism Determination of 10 Proprietary Chinese Medicines for Children by Plate Culture or Membrane Filtration

**DOI:** 10.1155/2022/6382676

**Published:** 2022-05-18

**Authors:** Hong Cai, Danchun Jia, Yuan Ke

**Affiliations:** Shangluo Institute for Drug Control, Shangluo, China

## Abstract

**Objective:**

This study attempted to verify the applicability of the microbial limit test (plate culture and membrane filtration) for 10 proprietary Chinese medicines for children.

**Methods:**

In this study, we collected 10 proprietary Chinese medicines for children as study objects and performed plate culture and membrane filtration to calculate the colony-forming unit (cfu) of microorganisms in these medicines and verify its applicability in objectionable microorganisms.

**Results:**

It was found that the recovery rate of microorganisms including *Staphylococcus aureus*, *Bacillus subtilis*, *Pseudomonas aeruginosa*, *Candida albicans*, and *Aspergillus niger* ranged from 70% to 150%. This verification was performed by plate culture or membrane filtration. Inspection for objectionable microorganisms (*Escherichia coli*, *Salmonella paratyphi* B, and bile salt-tolerant Gram-negative bacteria) was applicable for most medicines.

**Conclusion:**

Microbial limit test is feasible for the determination of microorganisms in 10 proprietary Chinese medicines for children.

## 1. Introduction

An increasing incidence rate of acute upper respiratory tract infections in children under 5 years of age has been observed in recent years, and the course of disease lasts for a long time. Proprietary Chinese medicines for children are commonly used in clinical practice due to lack of specific antiviral drug for common cold [1]. The safety of proprietary Chinese medicines for children has always been a social concern as a result of characteristics of growth and development. Most proprietary Chinese medicines are compound agents containing a variety of substances with complex components, which have bacteriostatic efficacy leading to a decrease in accuracy of the microbial limit test [2, 3]. Therefore, the study on the applicability of the microbial limit test for children's proprietary Chinese medicines not only ensures the integrity and accuracy of the test method, but also provides theoretical support for its safe use to a certain extent [4, 5]. 10 proprietary Chinese medicines, including Xiao'er Ganmao granule, Xiao'er Jiegan granule, Xiao'er Huatan Zhike granule, Xiao'er Feire Kechuan granule, Xiao'er Chaigui Tuire granule, Xiao'er Chiqiao Qingre granule, Xiao'er Yanbian granule, Jinlian Qingre granule, Kanggan granule, and An'erning granule, with different antibacterial components, are commonly given to children for cold [6, 7]. In this study, plate culture and membrane filtration were carried out to verify the applicability and accuracy of the microbial limit test in 10 children's proprietary Chinese medicines, which provided clinical value for acute upper respiratory tract infections in children.

## 2. Materials and Methods

### 2.1. Microorganism Suspension Preparation Scheme

*Staphylococcus aureus* (CMCC(B)26003), *Bacillus subtilis* (CMCC(B)63501), *Pseudomonas aeruginosa* (CMCC(B)10104), *Escherichia coli* (CMCC(B)44102), and *Salmonella paratyphi* B (CMCC(B)50094) were individually cultured in the nutrient broth medium for 24 hours at a room temperature of 35°C, followed by the addition of concentration of 0.9% sterile sodium chloride (NaCl) solution (Tianjin Hedong Hongyan Reagent Factory, China). The suspensions of the first three bacteria and the last two bacteria were 1 × 10^4^ cfu/ml and 1 × 10^2^ cfu/ml, respectively. 0.9% sterile NaCl solution was added to *Candida albicans* (CMCC(F)98001) cultured at 25°C for 24 hours in the modified martin broth medium. The germ-containing quantity of the suspension was 1 × 10^4^ cfu/ml. *Aspergillus niger* (CMCC(F)98003) was cultured at 25°C for 7 days in the modified martin agar medium and washed with 5 ml of 0.9% sterile NaCl solution containing 0.05% concentration of polysorbate 80 for extracting the spore. The spore suspension containing 10^4^ cfu/ml was prepared with 0.9% sterile NaCl solution mixed with 0.05% polysorbate 80. All strains were purchased from China Institute for Food and Drug Control.

### 2.2. Arrangement of Sample Solution

A total of 10 test samples, as listed in Table 1, were prepared for sample solution. Tryptic soy broth (TSB) (Beijing SanYao Science & Technology Development Co., China) was added to each test sample (10g/sample), respectively, to gain the solution with a ratio of 1 : 10. This sample solution was diluted with sterile pH 7.0 NaCl-peptone buffer for the preparation of the solution in the proportion of 1 : 10, 1 : 50, and 1 : 100, respectively.

### 2.3. Microbial Limit Test for Medicines

The plate culture was used as the preferred method to calculate the colony-forming unit (cfu) of aerobe, mold, and yeast in each group. Study group of aerobe: 10 ml of (1 : 10 scale) the prepared sample solution was, respectively, placed in the germ-free test tube, and a total of 5 tubes of each solution are available. The addition of the suspension of aerobes with 0.1 ml, including *Staphylococcus aureus*, *Pseudomonas aeruginosa*, *Bacillus subtilis*, *Candida albicans*, and *Aspergillus niger*, was performed to each test tube to obtain a solution with germ content of no more than 100 cfu/ml. Each of above mixed solutions with 1 ml and tryptic soy agar (TSA) (Beijing SanYao Science & Technology Development Co., China) with 20 ml were put together successively in the two germ-free plates for 48–72 h culture at 30–35°C.

Study group of mold and yeast: the solution (sample solution mixed with suspension of *Candida albicans* and *Aspergillus niger*) was prepared according to the above method, followed by 48–72 h culture in 20 ml of Sabouraud Dextrose Agar (SDA) (Beijing SanYao Science & Technology Development Co., China) at 20–25°C using 1 ml concentration of the mixed solution.

Microorganism group: 20 ml of TSB was added into 0.1 ml of suspension of 5 aerobes, respectively, keeping germ content of no more than 100 cfu/ml. It was cultured at 30–35°C for 48–72 h. As for mold and yeast, 20 ml of SDA was used to culture 0.1 ml of *Candida albicans* and *Aspergillus niger* suspensions individually. The germ-containing quantity was more than 100 cfu/ml. The culture conditions were set as 20–25°C for 48–72 h. Sample group: 10 ml of each sample solution (1 : 10 scale) was cultured in nutrient agar with 20 ml for 48–72 h.

Membrane filtration was applied to calculate the cfu of each group in the absence of recovery rate no more than 70%. The specific method of the study group was as follows: 1 : 10 scale of 10 ml of sample solution was mixed with 0.1 ml of microorganism suspension to gain the solution with no more than 100 cfu/ml, followed by filtration rinse of 1 ml of the mixed solution using 100 ml of pH 7.0 NaCl-peptone buffer. The membrane was filtered by 100 ml of pH 7.0 NaCl-peptone buffer 5 times. The membrane with microorganisms upward was stuck to the TSA plate for culture for 3 days at 30–35°C or 20–25°C. The preparation and determination of the microorganism group and sample group were performed according to the above-mentioned method.

### 2.4. Recovery Rate Calculation

Three parallelism tests were conducted for each group and their recovery rate was calculated. Recovery rate = ((average cfu of the study group − average cfu of the sample group)/average cfu of the microorganism group) × 100%. If the recovery rate is no less than 70% in the three parallelism tests, it shows that the counting methods of microorganisms and the proportion of the sample solution were verified.

### 2.5. Objectionable Microorganism Inspection

Bile salt-tolerant Gram-negative bacteria: it was mixed with each sample solution (1 : 10 scale), respectively, and cultured at 20–25°C for 2 h. 1 mL of the mixed solution was incubated in 10 ml of Enterobacteria Enrichment Broth Mossel with addition of 1 ml (10^2^ cfu/mL) of *Escherichia coli* and *Pseudomonas aeruginosa* suspension at 30–35°C for 24 h, followed by another culture with violet red bile glucose agar for 24 h at 30–35°C.

*Escherichia coli*: 10 mL of each sample solution (1 : 10 scale) and 1 mL of *Escherichia coli* suspension (10^2^ cfu/mL) were added to 100 mL TSB for incubation at 30–35°C for 18–24 h, respectively, and then 1 mL of the above mixed solution was blended with 100 mL of MacConkey Broth (MCB) for 18–24 h at 42–44°C. Streaking inoculation was performed with MacConkey Agar for 18–24 h at 30∼35°C on the solution incubated with MCB.

*Salmonella paratyphi* B: 100 mL TSB containing 1% polysorbate 80 was applied to culture 10 ml of each sample solution blended with 1 mL of *Salmonella paratyphoid* B suspension containing 10^2^ cfu/mL germs. It was placed at 30–35°C for 18–24 h. 0.1 mL of the solution was put into 10 mL of Rappaport Vassiliadis Salmonella Enrichment Broth (RVSEB) for 18–24 h at 30–35°C. Next, the solution cultured with RVSEB was streaked on Xylose Lysine Desoxycholate Agar for 18–48 h at 30–35°C.

## 3. Results

### 3.1. Determination of Aerobes in Medicines by Microbial Limit Test

The results in Table 2 showed that aerobes can be examined in Xiao'er Ganmao granule (G1), Xiao'er Feire Kechuan granule (G4), Xiao'er chaigui antipyretic granule (G5), and Xiao'er Yanbian granule (G7) using plate culture with 1 : 10 scale of the sample solution. Plate culture with 1 : 50 scale of the sample solution was applicable for the examination of *Pseudomonas aeruginosa* and *Bacillus subtilis* in Xiao'er Jiegan granule (G2), for the determination of *Staphylococcus aureus*, *Bacillus subtilis*, *Candida albicans*, and *Aspergillus niger* in Xiao'er Huatan Zhike granule (G3), for the measurement of *Bacillus subtilis* in Jinlian Qingre granule (G8), for inspection of *Staphylococcus aureus* in Kanggan granule (G9) and Xiao'er douqiao Qingre granule (G6), and for the detection of *Pseudomonas aeruginosa* in An'erning granule (G10) and Xiao'er douqiao Qingre granule (G6). *Bacillus subtilis* in G6 can be only inspected by membrane filtration.

### 3.2. Examination of Mold and Yeast in Medicines by Microbial Limit Test

As shown in Table 3, the data indicated that *Candida albicans* in Xiao'er Huatan Zhike granule (G3) can only be detected by plate culture when the sample solution was arranged in the proportion of 1 : 50. 1 : 10 scale of sample solution along with plate culture was suitable for mold and yeast's detection of the rest samples.

### 3.3. Inspection for Objectionable Microorganisms in Medicines

The results (Table 4) revealed that *Escherichia coli* can be detected in all medicines when the solution was incubated in 100 mL of TSB. 10 ml of Enterobacteria Enrichment Broth Mossel was applicable for determining bile salt-tolerant Gram-negative bacteria in medicines G1, G3, G6, G9, and G10. *Salmonella paratyphi* B in medicines G1, G3, G4, G6, G9, and G10 can be examined using 100 mL of TSB containing 1% polysorbate 80.

## 4. Discussion

Acute upper respiratory tract infections including common cold, rhinosinusitis, pharyngitis, tonsillitis, and otitis media are responsible for 87.5% of the total episodes of respiratory infections, resulting in huge health care costs annually [8]. Viruses are the main cause for the majority of acute upper respiratory tract infections. Over-the-counter drugs are not recommended for common cold in children younger than six years [9]. The earliest use of proprietary Chinese medicines can be traced back to 3000 years ago, and it was recorded in an ancient medical book which described many dosage forms, including pills, tablets, yeast, Baijiu, ointments, soups, and powders [2]. Proprietary Chinese medicines for children with upper respiratory tract infections are particularly prevalent in recent years. Therefore, ingredients of proprietary Chinese medicines are particularly important for children. In this study, we focused on microorganism detection in proprietary Chinese medicines. The results of this study showed that weak bacteriostasis was found in these 10 proprietary Chinese medicines commonly used in clinical practice for children. Plate culture was applicable for the calculation of total number of most aerobes when 1 : 10 or 1 : 50 scale of the sample solution was prepared. Bacillus subtilis in Xiao'er Chiqiao Qingre granule can only be determined by membrane filtration (1 : 100). The total number of molds and yeasts except for *Candida albicans* in Xiao'er Huatan Zhike granule can be checked by plate culture with a ratio of 1 : 10. Although some proprietary Chinese medicines for children contain ingredients with obvious bacteriostatic effects, the experimental results in our study revealed that these 10 proprietary Chinese medicines for children have little antibacterial effect, which proved that its content of active ingredients (g or mL) may be lower. In this study, microbial limit test for detection of microorganisms in 10 proprietary Chinese medicines was verified. Our data suggested that microbial limit test is an accurate and reliable method, which provided theoretical support for the applicability of the microbial limit test to similar proprietary Chinese medicines. However, further study should be performed to find out which culture medium and specific method are applicable for detecting objectionable microorganisms including bile salt-tolerant Gram-negative bacteria and *Salmonella paratyphi* B in medicines such as G2, G4, and G5.

## Figures and Tables

**Table 1:** Production information of 10 proprietary Chinese medicines for children.

Sample	Batch no.	Specification	Manufacturer
Xiao'er Ganmao granule (G1)	20031741	12 g/bag	Xi'an Bicon Pharmaceutical Group Co., Ltd.
Xiao'er Jiegan granule (G2)	21105017	2.5 g/bag	Freda Pharmaceutical Co., Ltd.
Xiao'er Huatan Zhike granule (G3)	201102	5 g/bag	Sichuan Caihong Pharmaceutical Co., Ltd.
Xiao'er Feire Kechuan granule (G4)	210309	4 g/bag	Huluwa Pharmaceutical Co., Ltd.
Xiao'er Chaigui Tuire granule (G5)	A20210514	4 g/bag	Guizhou Bailing Pharmaceutical Co., Ltd
Xiao'er Chiqiao Qingre granule (G6)	2106024	2 g/bag	Jichuan Pharmaceutical Co., Ltd.
Xiao'er Yanbian granule (G7)	20200308	4g/bag	Panlong Pharmaceutical Co., Ltd.
Jinlian Qingre granule (G8)	191129	2.5 g/bag	Qiyuan Pharmaceutical Co., Ltd.
Kanggan granule (G9)	210422	4 g/bag	Good Doctor Pharmaceutical Group
An'erning granule (G10)	2190703	3 g/bag	Jinhe Tibetan Pharmaceutical Co., Ltd.

**Table 2:** Recovery rate of aerobes in medicines (%).

Sample	Method	*Staphylococcus aureus*	*Pseudomonas aeruginosa*	*Bacillus subtilis*	*Candida albicans*	*Aspergillus niger*
G1	Plate culture (1 : 10)	100/90/100	90/80/80	100/100/100	90/90/80	0.9/0.9/0.9
G2	Plate culture (1 : 10)	80/80/90	40/30/30	20/30/20	80/80/80	70/80/80
	Plate culture (1 : 50)		130/120/120	90/100/100		
G3	Plate culture (1 : 10)	40/30/40	130/120/120	40/30/40	—	—
	Plate culture (1 : 50)	100/100/90		70/80/70	80/80/80	90/90/90
G4	Plate culture (1 : 10)	100/100/100	140/150/140	120/120/100	80/80/90	9080//90
G5	Plate culture (1 : 10)	100/90/90	110/110/110	130/120/110	80/80/80	90/90/110
	Plate culture (1 : 10)	—	30/30/30	—	80/80/80	90/90/110
G6	Plate culture (1 : 50)	70/75/70	90/80/90	30/30/30		
	Plate culture (1 : 100)			40/30/40		
	Membrane filtration (1 : 100)			80/70/70		
G7	Plate culture (1 : 10)	100/100/90	150/140/140	72/75/70	90/80/90	100/90/110
G8	Plate culture (1 : 10)	70/70/80	140/130/130	20/30/30	90/90/80	90/90/90
	Plate culture (1 : 50)			80/73/78		
G9	Plate culture (1：10)	40/30/40	130/130/130	75/70/70	100/90/90	100/110/90
	Plate culture (1 : 50)	100/90/90				
G10	Plate culture (1 : 10)	90/90/90	30/40/30	80/70/80	90/90/80	100/90/90
	Plate culture (1 : 50)		110/140/110			

**Table 3:** Recovery rate of mold and yeast in medicines (%).

Sample	Method	*Candida albicans*	*Aspergillus niger*
G1	Plate culture (1 : 10)	70/80/80	90/80/90
G2	Plate culture (1 : 10)	70/70/70	72/70/75
G3	Plate culture (1 : 10)	—	70/70/70
	Plate culture (1 : 50)	90/80/90	
G4	Plate culture (1 : 10)	70/70/80	80/80/80
G5	Plate culture (1 : 10)	70/70/70	100/90/90
G6	Plate culture (1 : 10)	90/80/80	110/100/100
G7	Plate culture (1 : 10)	71/75/70	100/90/100
G8	Plate culture (1 : 10)	80/80/80	100/90/100
G9	Plate culture (1 : 10)	90/90/90	100/90/90
G10	Plate culture (1 : 10)	70/70/80	75/70/75

**Table 4:** Objectionable microorganism inspection in medicines (medium volume (mL)).

Sample	Bile-salt-tolerant Gram-negative bacteria	*Escherichia coli*	*Salmonella paratyphi* B
G1	10	100	100
G2	—	100	—
G3	10	100	100
G4	—	100	100
G5	—	100	—
G6	10	100	100
G7	—	100	—
G8	—	100	—
G9	10	100	100
G10	10	100	100

## Data Availability

The data supporting the findings of this study are included within the article.
